The article "Oral Pemphigus Vulgaris" was published in 2021. Journal: Cureus.

# Oral Pemphigus Vulgaris

**DOI:** 10.7759/cureus.18005

**Published:** 2021-09-15

**Authors:** K Subadra, Sathasivasubramanian S, Aravind Warrier S

**Affiliations:** 1 Oral Medicine and Radiology, Sri Ramachandra Institute of Higher Education and Research, Chennai, IND

**Keywords:** desmoglein, pemphigus vulgaris, bullae, tzanck test, triamcinolone acetonide, mycophenolate mofetil

## Abstract

Pemphigus is a chronic mucocutaneous autoimmune disease with the clinical feature of blisters that initially appear in the oral cavity and later in the skin. The dental professionals play an important role in diagnosing the disease. Early diagnosis and treatment determine the course and prognosis of the disease. Systemic corticosteroids continue to be the standard therapy for pemphigus vulgaris (PV). Management of PV involves prolonged use of steroids to control the disease and prevent relapses, but associated adverse events constantly remain a great challenge. Regular periodic clinical evaluation of patients with pemphigus on steroids is mandatory. This article describes a case of a 50-year-old woman with multiple chronic ulcers in the oral cavity in whom the diagnosis of PV was made and treated. The case study is followed by a review of the literature including etiology, pathogenesis, clinical features, as well as the various diagnostic criteria and the therapeutic options of PV.

## Introduction

Pemphigus is a life-threatening autoimmune disorder characterized by bulla and ulcers in the mucocutaneous region [1]. Pemphigus vulgaris (PV), pemphigus vegetans, pemphigus erythematosus, pemphigus foliaceus, and paraneoplastic pemphigus are the various types of pemphigus [2]. Pemphigus vegetans belong to the group of PV, pemphigus erythematosus to pemphigus foliaceus respectively. The lesion involves the superficial granular cell layer in pemphigus foliaceus; in the case of PV, it occurs deeper in the supra-basal cell layer [1]. Among these groups, the common variant which develops oral lesions as one of the early manifestations in 50% of the cases is PV [3]. Oral involvement appears to be uncommon in other variants such as pemphigus erythematosus and pemphigus foliaceus [1]. The progressive course of the disease includes loss of body fluids, proteins, and secondary infection which may lead to sepsis and cardiac failure. The mortality rate of this disease was high within two years of diagnosis, before the introduction of systemic corticosteroids. The underlying pathogenesis responsible for the development of the intraoral lesion was brought out by binding of IgG autoantibodies to transmembrane glycoprotein adhesion proteins, desmoglein 3 on keratinocyte cell surfaces [4]. As the oral mucosa is often the first affected site in PV, oral physicians play a critical role in diagnosing and managing oral lesions [3]. Subsequently, the real challenge remains in obtaining rapid remission as early as possible to reduce the rate of relapse and side effects associated with treatment agents such as steroids and immunosuppressive agents [5]. This article describes a case of oral PV and its management. The case study is followed by a review of the literature on etiology, pathogenesis, clinical features, as well as the various diagnostic criteria and the therapeutic options of PV.

## Case presentation

A 50-year-old female Asian patient reported to the Department of Oral Medicine and Radiology with a two month history of multiple painful oral ulcers with difficulty in eating and swallowing solid food . Initially she noticed a bullae in her left buccal mucosa which was initially small and later involved the entire oral cavity. The patient had medical consultation and was prescribed topical medication and vitamin supplements with no relief. Her medical and family history was not significant. The patient showed no signs of skin and other mucosal involvement. Intraoral examination revealed a large shallow irregular ulcer, about 4 cm x 4 cm in diameter on the left buccal mucosa. The ulcer was round in shape with irregular margins and an erythematous halo. The base of the ulcer was covered with yellowish white pseudomembrane interspersed with erythematous area. Multiple irregular shallow ulcers were observed in the right buccal mucosa, lower labial mucosa, ventral surface, and the right and left lateral border of the tongue. Multiple pin-point isolated ulcers were evident in the soft palate (Figures 1-3).

**Figure 1:** Multiple shallow ulcers with erythematous halo and tissue tags in the right (A) and left (B) buccal mucosa; soft palate (C) and lower labial mucosa (D).

**Figure 2:** Ruptured bullae in the right (A) and left (B) lateral border of the tongue.

**Figure 3:** Ventral surface of the tongue. Multiple ruptured bullae with erythematous halo in the ventral surface of the tongue.

The ulcers were tender, with a yellowish white pseudomembrane on the floor that peeled off leaving an erythematous area that bled on palpation. Correlating the history of bullae and the clinical features of multiple chronic oral ulcers, the fragility of the oral mucosa (Nikolsky’s sign), the provisional diagnosis of oral PV was made. Since chronic oral ulcers are common in conditions of erosive lichen planus, mucous membrane pemphigoid, bullous pemphigoid, and major variants of pemphigus paraneoplastic pemphigus and pemphigus foliaceous were considered in the clinical differential diagnosis. The erosive form of lichen planus (LP) frequently presents with the characteristic feature called Wickham’s striae, along with erosions. Mucous membrane pemphigoid is more common in females with intact vesicles of the gingival or other mucosal surfaces. The erosions spread more slowly than PV. Bullous pemphigoid occurs chiefly in adults over the age of 60, oral lesions are smaller, form more slowly, and are less painful than those seen in PV, and the extensive labial involvement seen in pem­phigus is not present. Paraneoplastic pemphigus is a severe variant of pemphigus that is associated with erosions in the mucous membrane and the skin associated with an underlying neoplasm. Mucosal involvement is uncommon in foliaceus and erythematous forms of the disease [1]. The smear was taken from the right buccal mucosa and subjected for exfoliative cytology and the smear showed acantholytic cells, a few normal squamous epithelial cells along with mixed inflammatory cells chiefly lymphocytes and neutrophils suggestive of pemphigus (Figure 4). Incisional biopsy was performed on the perilesional site of the right buccal mucosa and was subjected for histopathological investigation.

**Figure 4:** Tzanck smear. Smear reveals acantholytic cells

Histopathology in the present case was characterized by stratified squamous epithelium with intraepithelial bullae containing acantholytic cells and characteristic tombstone appearance, connective tissue with mixed inflammatory cells chiefly plasma cells and lymphocytes and fibro adipose tissue in the deeper section, suggestive of PV with secondary infection (Figure 5).

**Figure 5:** Incisional biopsy. Low-power photomicrograph shows intraepithelial cleft and underlying connective tissue with chronic inflammatory cells (hematoxylin-eosin 10x).

Correlating the clinical and the histopathological features, a final diagnosis of oral PV was made. The patient was started on oral prednisolone at an initial dose of 20 mg, in divided doses of 5 mg, four times a day, along with topical application of triamcinolone acetonide oral paste 0.1%, three times a day after meals for about one hour. In addition, the patient was given hexidine mouth rinse for oral prophylaxis and clotrimazole oral paint 1% twice a day after topical application of steroids for an hour to prevent secondary fungal infection for one week. Treatment was continued for another week with the same dosage since there were few lesions present. After two weeks the dosage was tapered to 10 mg, in divided doses of 5 mg, two times daily for another two weeks. At the end of the fourth week, prednisolone was decreased to 5 mg single dose for two weeks. The patient got recovered. She was periodically reviewed once a month, over a period of seven months, with no recurrence of oral lesions (Figures 6-8).

**Figure 6:** Completely healed lesions in right (A) and left (B) buccal mucosa; soft palate (C) and lower labial mucosa (D).

**Figure 7:** Completely healed lesions in right (A) and left (B) lateral border of the tongue.

**Figure 8:** Ventral surface of the tongue. Completely healed lesions.

## Discussion

Pemphigus vulgaris is one of the rare autoimmune disorders with intraepithelial blisters involving the skin and mucous membrane. The term pemphigus originated from the Greek word Pemphix (bubble or blister). It is a very rare disease with the prevalence of 0.1-0.5 cases per 100,000 inhabitants per year [6-7]. According to the literature it is the most prevalent in the fourth to sixth decade of life, showing female predominance with male to female ratio of about 1:2 [7]. 

The etiology of PV is uncertain. The pemphigus group of diseases are classified as autoimmune diseases since they are manifested by the development of autoantibodies against intercellular substances. Viral infection may also act as predisposing factor in the production of autoantibody [8]. It also can be aggravated by other environmental factors such as foods (garlic), infections, neoplasms, and drugs. Most commonly, drugs that belong to the thiol group, such as captopril, penicillamine and rifampicin, have been associated with the disease [9-10]. It is more common in patients of Mediterranean, Jewish, and Asian (particularly Indian and Japanese) descent [3, 7, 11]. Increased susceptibility to Class II alleles of human leukocyte antigen was also evident. However thorough medical, personal, and drug history was made in our case to rule out the possibility of infection and drugs as the initiating factor. Furthermore the onset of the lesions in our case did not corelate with the above-mentioned etiological factors.

 Pemphigus vulgaris results from an autoantibody reaction, when serum IgG antibodies are directed against desmosomes on the keratinocytes in the cell membrane [9]. Desmosome molecules particularly desmoglein3 and desmoglein1 belong to the cadherin family, mainly responsible for holding the epithelial cells together [9]. In early stage PV with oral lesions, autoantibodies develop against desmoglein3. In advanced stages, with both skin and oral lesions, antibodies were present against both desmoglein1 and desmoglein3 [9]. This is because desmoglein3 is predominantly expressed in oral mucosa while both desmoglein1 and desmoglein3 are expressed in skin [10]. The primary serum antibodies IgG type is mainly responsible for development of PV, IgG1 indicates remission phase and IgG4 the active phase of the disease respectively [11-12]. 

In 70%-90% of PV cases, early manifestation of the disease is on the oral mucosa consistent with our case [9]. Even though the lesions appear to involve the entire oral cavity, the most common sites are the buccal mucosa, tongue, palate, and lower lip, most frequently located in areas subjected to friction [9]. In our case the lesions were found in the same site as per literature. Bulla in the oral mucosa have a very thin roof and readily rupture due to oral trauma, giving rise to multiple chronic painful bleeding ulcers and erosions as shown in Figure 1 [3]. According to Dagistan et al., ulcers may also develop on the mucosa of the eyes, nose, pharynx, larynx, esophagus, genital mucosa besides oral mucous membrane [13]. The major subjective complaints are increased salivation and difficulty in chewing and swallowing, as in our patient [14]. Good prognosis with better quality of life will be provided to the patient with early detection and treatment of oral lesions. PV can be dangerous if left untreated, something like fungal infection, loss of fluid and protein [9].

The diagnosis of PV is generally based on three independent sets of criteria such as clinical features, histopathology, and immunological tests [12]. According to Davenport et al. oral manifestations of hemorrhagic bullae or shallow irregular ulcers, with characteristic finding of whitish superficial covering representing collapsed bullae, rapidly rupturing bullae mainly in the sites of buccal mucosa, palate, tongue, lips is consistent with PV [3, 9, 15]. Nikolsky's sign is an important clinical diagnostic criterion which is done by pressing the lesion in the skin with the finger for the appearance of a new blister. Although accuracy about sensitivity and specificity of this test has been in question [9,16], it has been a very useful clinical diagnostic tool and pathognomic of PV with specificity of about 96.3% in the oral lesions [17]. Generally following the clinical diagnosis, confirmation of the lesion is provided by histological findings.

 Histopathologically PV is characterized by intraepidermal acantholysis, with basal keratinocytes still attached to the basement membrane zone assuming a characteristic tombstone-like morphology [18]. In our case, a biopsy of intraoral lesions was obtained and the tissue was stained with hematoxylin- eosin and the histological report represents the principle features of stratified squamous epithelium with intraepithelial bullae containing acantholytic cells and characteristic tombstone appearance consistent with the literature. Other diagnostic examination includes direct immunofluorescence test of perilesional mucosa for detection of IgG, IgM, IgA, and C3 protein. Blood tests such as indirect immunofluorescence and enzyme-linked immunosorbent assay for autoantibodies against desmoglein glycoproteins are carried out. Tzanck smear to detect acantholytic cells, is useful in lesions of the oral mucosa. In addition, techniques such as immunoblot analysis and immunoprecipitation tests were done when the diagnosis remains uncertain [9, 13, 16].

Hrabovska et al. compared and analyzed the importance of both histopathology and immunofluorescent examination individually in the tissue of PV. He found both histopathology and direct immunofluorescent examinations were equivalent in the diagnosis of PV. He concluded that direct immunofluorescence assay is required only in establishing the diagnosis of PV, especially when the clinical and histopathology findings are not clear [19]. In our present case, clinical and histopathology features were consistent with the criteria hence direct immunofluorescence was not opted. Moreover, false negativity of direct immunofluorescence due to the selection of biopsy site, treatment status, technical errors and financial constraints were the main limitation [20]. Indirect immunofluorescence tests are performed to assess the titer of circulating autoantibodies, to be an index of disease severity more suitable for determining the success of treatment [21]. However, assessing the titer of circulating antibodies is costly and it is used mainly for evaluating the severity of the disease and for the treatment plan.

 However other dermatological disorders associated with large bullae in the oral mucosa considered as differential diagnosis should be ruled out. Pemphigus vegetans is very rarely characterized by verruciform and papillomatous vegetating and/ or pustular lesions of the periorificial regions [22]. In our case there is no evidence of periorificial lesions. In paraneoplastic pemphigus, clinical features include cheilitis and/or ulcerative stomatitis, chronic painful erosions with dysphagia. Moreover, the lesion can precede the malignancy. Its histopathological features are polymorphic. Bullous lesions have supra-basal acantholysis with dyskeratosis with a scattered inflammatory infiltrate. A lichenoid interface dermatitis is more frequently observed in maculopapular lesions [22-23]. Clinically mixed maculopapular and bullous lesions show both acantholysis and lichenoid interface dermatitis [24]. Clinically pemphigus foliaceous represents more of skin lesion with no mucosal involvement; biopsy report shows more superficial, subcorneal acantholysis [22-23]. Our present case did not represent any cutaneous lesions and systemic manifestation over a period of seven month of follow up. Our histological findings did not represent dyskeratosis and acantholysis in the stratum corneum. 

The main aim of the treatment is to induce disease remission. PV is generally managed with topical, oral, and intralesional corticosteroids. Systemic corticosteroids have been used as the cornerstone of management for PV since the time of their approval in the 1950s. Mechanism of action of corticosteroids is through interaction with the cytoplasmic corticosteroid receptor, resulting in upregulation of the expression of anti-inflammatory proteins and downregulation of the expression of pro-inflammatory proteins, interleukin (IL)-2 [25]. IL-2 reduces both B-cell clone expansion and autoantibody synthesis. The decrease in IL-2 also suppresses cell-mediated immunity and reduces T-cell proliferation. Hence the corticosteroid therapy results in anti-inflammatory, immunosuppressive, antiproliferative, and vasoconstrictive effects [26]. 

Almugairen et al., stated that, in patients without complications, the disease activity is controlled within several weeks by oral systemic corticosteroid, but needs a month for complete remission on minimal therapy and often needs more months or years for complete remission off therapy [27]. There are inadequate guidelines to ascertain the optimal dose of corticosteroids. European Dermatology Forum and European Academy of Dermatology and Venereology recommended administration of a higher prednisolone dose (up to 2 mg/kg) if the control of the disease is not achieved with an initial dose of prednisolone of 0.5 mg-1.5 mg/kg/d within two weeks [22]. In the present case consistent with the literature we started on a low dose to reduce the side effect. Ratnam et al., did a randomized control trial in patients who were put through both high- and low-dose of corticosteroids in a period of five years and found out that there was no marked difference in the period of healing and recurrence rates [28]. Systemic corticosteroids can be combined with an immunosuppressive adjuvant, particularly when complications such as hypertension, diabetes mellitus, and osteoporosis, are expected due to prolonged use of corticosteroid therapy(>4 months) [22].

Furthermore combined or single use of immunosuppressants such as azathioprine, mycophenolate mofetil, dapsone, methotrexate, cyclophosphamide, and cyclosporine should be considered as second drug of choice in case of contraindications to glucocorticoids or its side effects related to prolonged duration of therapy (>4 months). If the disease is severe and progresses rapidly, not responding to standard oral corticosteroids, immunosuppressants pulse therapy with high dose of IV methylprednisolone or cyclophosphamide, plasmapheresis, and intravenous immunoglobulin (IVIG) may be required [12]. Novel improvement in medical management that involves biologics such as infliximab, especially rituximab and intravenous immunoglobulin (IVIG), reveals that it contributes to very good effect in case of refractory PV [5]. 

As a complement to treatment, intralesional injections of corticosteroids (triamcinolone acetonide) may be beneficial for isolated lesions of oral mucosa, lips, and skin. Topical application of potent corticosteroids (clobetasol propionate), or calcineurin inhibitors directly to the lesions and combination of systemic therapy with typical oral corticosteroids (such as triamcinolone acetonide gel) may be beneficial in oropharyngeal erosions. Following measures like topical application of local anesthetic gel, administration of analgesics such as (paracetamol, metamizole, and opioids), maintaining good oral hygiene using antiseptic (chlorhexidine) mouthwashes, periodontal treatment, advising a soft diet without irritants, evaluating prosthetic restorations, help of a dietician or a nutritionist, nutrition management in case of malnutrition and applying anti-candida therapy on long-term corticosteroid treatments can be done to improve the wellbeing of patients [22]. Since pemphigus shows a chronic (relapsing) course it requires close monitoring of clinical symptoms and of potential side-effects related to chronic immunosuppressive treatment. Thus, a multidisciplinary approach is often essential.

Complete healing of lesions often requires a period of one to three months. In case of progressive reduction of oral corticosteroid treatment, gradually taper steroids as early as possible, once disease control is reached, or up to the end of consolidation phase. Prednisolone is tapered by 25% biweekly (at <20 mg more slowly). During the gradual reduction of oral corticosteroid regimen, if there is a recurrence of <3 lesions return back to previous dose. In case of relapse, re-increase oral corticosteroid treatment, and return two steps back in last dose till control of the lesions is obtained in a period of two weeks, then resume gradual reduction of systemic corticosteroids. If disease control is not reached go back to initial dose. Especially in early-stage relapse, occurring despite of continued high-dose corticosteroid, add an immunosuppressant, to the regimen. In case of relapse, if oral corticosteroids are already combined with an immunosuppressant, consider replacement in ﬁrst-line or second line immunosuppressant adjuvants [22].

## Conclusions

Pemphigus vulgaris is a rare cause of chronic ulceration of the oral mucosa. The mouth may be the only site of involvement for a year and it can lead to delayed diagnosis and inappropriate treatment of potentially fatal disorder. In the present case, due to early diagnosis, we could control the disease with lower doses of medication. The management of PV continues to be challenging. Henceforth early and accurate diagnosis of the lesion helps to initiate the treatment earlier thereby providing patient comfort, preventing the severity of the disease, hence as oral physician we play an inevitable role. Corticosteroids remain the gold standard treatment. Discovery of new medications and advanced me0dical management has markedly reduced the mortality rate of PV. Research advances have expanded the light on discovering the most effective steroid-sparing agent against PV, despite proof is uncertain. However, multicenter studies need to be incorporated to establish the common definitions and guidelines, and to determine optimal multistep algorithmic treatment regimens of pemphigus, contribute in reducing the duration of therapy and good standard of life for the patients.
